# Clinical Observation on Therapeutic Effect of Electroacupuncture Combined with Diclofenac Sodium in Treatment of Acute Gouty Arthritis: A Randomized Controlled Study

**DOI:** 10.1155/2022/3363064

**Published:** 2022-08-29

**Authors:** Lumin Liu, Ping Yin, Junwei Hu, Xu Li, Yuelai Chen

**Affiliations:** Longhua Hospital Affiliated to Shanghai University of Traditional Chinese Medicine, Shanghai 200032, China

## Abstract

**Objective:**

To observe the clinical effect of electroacupuncture (EA) combined with diclofenac sodium (DS) in the treatment of acute gouty arthritis (AGA).

**Methods:**

Patients with AGA were randomly divided into three groups: the EA + DS treatment group (i.e., EA + DS group), the low-dose DS treatment group (i.e., low-dose DS group), and the conventional-dose DS treatment group (i. e., conventional DS group). Patients in the low-dose DS group took 50 mg of DS sustained-release capsules once a day. Patients in the conventional DS group took 100 mg of DS sustained-release capsules once a day. Patients in the EA + DS group were treated with EA three times in 7 days combined with 50 mg of DS sustained-release capsules once a day. For all the three groups, 7 days were regarded as a course of treatment. Outcome indicators included pain visual analog scale (VAS), joint tenderness, joint swelling and activity limitation, and levels of inflammatory indicators (C-reactive protein (CRP)/white blood cells (WBC)/percentage of neutrophils (NE%)), level of serum uric acid (SUA), gout impact scale (GIS), and frequency of adverse reactions).

**Results:**

After a course of treatment, indicators regarding the VAS, joint tenderness, joint swelling, activity limitation, GIS, inflammatory indicators (CRP/WBC/NE%), and SUA were all improved (*P* < 0.05) with no adverse reactions in the EA + DS group. The EA + DS group performed better than the low-dose DS group in improving indicators regarding the VAS, joint tenderness, activity limitation, GIS, inflammatory markers (WBC/NE%), and SUA (*P* < 0.05). Similarly, the EA + DS group performed better than the conventional DS group in improving indicators regarding GIS, SUA, and adverse reactions (*P* < 0.05).

**Conclusion:**

EA combined with DS can improve AGA patients' joint pain and functional status, thus improving their quality of life. Moreover, this combined treatment can reduce the levels of inflammatory markers and SUA, leading to fewer adverse reactions in AGA patients.

## 1. Introduction

Gouty arthritis (GA) is a disease caused by the deposition of monosodium urate in joints due to disturbance of purine metabolism and/or decreased uric acid excretion. In the acute stage, GA is mostly manifested by sudden redness, swelling, heat, pain, and activity limitation of a single metatarsophalangeal joint (especially the first metatarsophalangeal joint), and the symptoms often involve other joints of the feet and the ankles [1].

Epidemiological surveys show that the prevalence of GA is increasing year-by-year [2]. The National Health and Nutrition Examination Survey found that between 2015 and 2016 there were 9.2 million adults diagnosed with GA in the United States [3]. In the United Kingdom, the prevalence of GA increased from 1.4% in 2005 to 2.5% in 2015 [4, 5]. GA has become the second-largest metabolic disease in China, with about 14 million people diagnosed every year [6]. During acute GA (AGA) attacks, the severe or unbearable pain can result in activity limitation, seriously affecting patients' physical and mental health as well as their quality of life [7, 8]. Besides, AGA imposes an economic burden on individuals and society [9].

In Western medicine, treatment of AGA is mainly based on drug therapy, including nonsteroidal anti-inflammatory drugs (NSAIDs), colchicines, and glucocorticoids [1]. Among them, NSAIDs are typically used as the first-line drugs, such as diclofenac sodium (DS) and indomethacin. Studies have shown that DS can improve joint pain and swelling, reduce levels of prostaglandin, interleukins, tumor necrosis factors, and other inflammatory factors in patients with AGA [10]. However, the main concern for the clinical practice of DS is the adverse reactions. A study on facet joint pain showed that adverse reactions, including nausea, vomiting, diarrhea, edema, and anaphylaxis, occurred during the administration of DS, the occurrence of which was higher in patients treated with higher doses [11]. Due to these adverse reactions, patients may stop taking the drugs. Therefore, an effective and multimodal therapy with fewer adverse reactions is urgently needed.

As a modern acupuncture therapy, electroacupuncture (EA) has been widely recognized for its analgesic effect [12, 13]. Preliminary studies have confirmed the effectiveness of EA in the treatment of AGA, including improvement of pain, swelling, and activity limitation [14]. However, the existing randomized controlled trials (RCTs) published might be biased or of low quality. For example, generation and concealment of allocation sequence and blind implementation were not mentioned or properly carried out in some of these existing RCTs. In addition, none of these RCTs explored whether EA combined with NSAIDs could reduce the dosage of analgesic drugs and its adverse reactions during AGA treatment. Considering these limitations in existing RCTs, the current research was designed to provide a more effective clinical solution for AGA treatment with fewer adverse reactions.

## 2. Methods

This RCT was conducted in Yueyang Integrated Traditional Chinese and Western Medicine Hospital affiliated to Shanghai University of Traditional Chinese Medicine in Shanghai, China, from October 2020 to February 2021. The trial was registered at the Chinese Clinical Trial Registry (ChiCTR2000039458) and approved by the Chinese Ethics Committee of Registering Clinical Trials (ChiECRCT20200279). Written informed consent was obtained from all participants. The RCT was carried out following the flow diagram shown in Figure 1.

### 2.1. Inclusion and Exclusion Criteria

The inclusion criteria are as follows:

- Those aged between 35 and 70 years
- Male patients
- The symptoms meet the GA diagnostic criteria jointly formulated by the American College of Rheumatology (ACR) and the European League Against Rheumatism (EULAR) in 2015
- The symptoms comply with the diagnostic criteria of AGA in the “Traditional Chinese Medicine Syndrome Diagnosis and Efficacy Criteria” [15] promulgated by the State Administration of Traditional Chinese Medicine in 2012 and belong to the dampness-heat amassment pattern
- The symptoms involve unilateral first metatarsophalangeal joint and/or foot (nonfirst metatarsophalangeal) joint and/or ankle joint
- The acute attack occurred within 24 hours when admitted to the hospital, and the visual analog scale (VAS) is greater than or equal to 4

The exclusion criteria are as follows:

- Patients allergic to NSAIDs
- Patients who had a pacemaker installed, allergic to metal, or had a severe fear of needles
- Patients who received acupuncture treatment within one week before treatment
- Patients who have used any drugs for the treatment of AGA within one month before treatment
- Patients with active gastrointestinal diseases or those who had peptic ulcers within 30 days before participating in this study
- Patients with primary severe diseases in the heart, brain, liver, kidney, hematopoietic system, or those with mental illness

### 2.2. Sample Size Calculation

According to the preliminary experimental results, the variation of VAS from baseline to treatment completion in the EA + DS group, conventional DS group, and low-dose DS group were 5.00 ± 0.38, 4.70 ± 0.82, and 3.60 ± 1.41, respectively. According to the calculation formula, $n=\varphi^{2}\left({\sum s_{i}^{2}/g}^{}\right)/\left(\sum {\left(\bar{X_{l}}-\bar{X}\right)}^{2}/\left(g-1\right)\right)$ [16], each group requires 25 cases (*α* = 0.05, *β* = 0.1). Considering the 15% dropout rate, each group requires 30 cases. Thus, a total of 90 cases are needed.

### 2.3. Randomization and Blinding

According to random numbers generated by SPSS 26.0 software, 90 patients were assigned to the EA + DS group, conventional DS group and low-dose DS group at a ratio of 1 : 1 : 1. All information regarding random sequence used for the grouping was sealed in a separate light-tight envelope, which could not be opened until each patient's enrollment. Criteria evaluation and clinical information collection of patients were performed by information collection personnel, and statistical data analyses were performed by specialized statisticians. The information collection personnel and statisticians were blinded to each other. Grouping was performed by special grouping personnel, and the grouping information was blinded to the information collection personnel and statisticians. Based on the characteristics of this study, patients and acupuncturists could not be blinded.

### 2.4. Clinical Grouping and Intervention Methods

#### 2.4.1. Low-Dose DS Group

Patients took DS sustained-release capsules (trade name: Yingtaiqing, 50 mg, produced by Simcere Pharmaceutical Co., Ltd., batch no. H20023856) orally, 50 mg each time, once per day. 7 days were regarded as a course of treatment.

#### 2.4.2. Conventional DS Group

The drug used and course of treatment was the same as above, except for those who took 100 mg of the capsules orally once per day.

#### 2.4.3. EA + DS Group

For the EA + DS group, patients were treated with EA once every three days (3 times in total), while at the same time, they were treated with DS the same as in the low-dose DS group, with 7 days as a course of treatment.

All acupuncture manipulations were performed by an acupuncturist with TCM qualification and rich experience. The patients received acupuncture treatments on the affected side at the Ashi, Dadu (SP2), Taichong (LR3), Taibai (SP3), Neiting (ST44), Sanyinjiao (SP6), Zusanli (ST36), and Yinlingquan (SP9) points. In order to prevent fainting during acupuncture treatment, the acupuncturist explained the procedures to the patients and comforted them during the treatment. The acupuncture would be avoided when the patients were hungry. The skins of the acupoints were disinfected with 75% alcohol, and then two types of acupuncture needles (Huatuo disposable sterile stainless steel acupuncture needles, Suzhou Huatuo Medical Equipment Co., Ltd.) were used for acupuncture treatment. Specifically, a 0.25^*∗*^25 mm needle was inserted straight into the Ashi (5–10 mm), SP2 (5–10 mm), ST44 (5–10 mm), LR3 (10–15 mm), and SP3 (10–15 mm) acupoints. A 0.25^*∗*^40 mm needle was inserted straight into the SP6 (20–25 mm), ST36 (20–30 mm), and SP9 (20–30 mm) acupoints. When directly inserted into the skin, the needle was manipulated clockwise and counterclockwise to obtain a sense of “Deqi,” which was then connected to the EA instrument (Huatuo G6805-II electroacupuncture instrument, Shanghai Medical Electronic Instrument Physiotherapy Branch), with LR3 and ST36 as a group and SP9 and SP6 as another group. For the EA, the wave was a continuous wave, the frequency was 2 Hz, and the current was 1–5 mA (to a degree when the skin is shaking slightly at the acupoints but the patient did not feel pain). The needles were kept in the acupoints for 30 minutes.

### 2.5. Outcome Indicators and Observation Time

Primary outcomes included VAS and its variation from baseline to treatment completion. Secondary outcomes included joint tenderness, joint swelling, activity limitation, gout impact scale (GIS) [17], levels of C-reactive protein (CRP), white blood cells (WBC), percentage of neutrophils (NE%), serum uric acid (SUA), and their variation from baseline to treatment completion. All these indicators were observed before treatments (i.e., baseline) and after treatments. In addition, adverse events and safety observation of EA were documented throughout the trial.

### 2.6. Data Analysis

SPSS 26.0 software was used for all data analyses. For intragroup comparisons, a paired-sample *t*-test was used for measurement data that conformed to a normal distribution, and otherwise, the Wilcoxon nonparametric test was used. For intergroup comparison, one-way ANOVA was used for measurement data that conformed to a normal distribution, and otherwise, the Kruskal–Wallis nonparametric test was used. The test standard was *α* = 0.05, and *P* < 0.05 was considered statistically significant.

## 3. Results

### 3.1. Demographics and Baseline Results

A total of 117 patients were screened in this study, and a total of 90 patients who met the inclusion criteria were finally included, with 3 patients dropping out during the treatment. The dropout reasons are shown in the flow chart (Figure 1). Thus, 87 cases were actually included in the study, including 28 cases in the low-dose DS group, 29 cases in the conventional DS group, and 30 cases in the EA + DS group. In general, there were no differences regarding age, body mass index (BMI), and disease duration among the three groups (*P* > 0.05). In terms of outcome indicators, there were no differences at baseline among the three groups (*P* > 0.05) (Table 1).

### 3.2. Indicators Like VAS, Joint Tenderness, Joint Swelling, and Activity Limitation

Intragroup analyses showed significant improvements regarding VAS, joint tenderness, joint swelling, and activity limitation after treatment compared to baseline in all three groups(*P* < 0.05). After treatment, VAS, joint tenderness, joint swelling, activity limitation, and their variation from baseline to treatment completion in the EA + DS group and conventional DS group were all lower than those in the low-dose DS group (*P* < 0.05), except for the variation of joint swelling. There were no differences regarding these indicators between the EA + DS group and the conventional DS group (*P* > 0.05) (Table 2).

### 3.3. GIS

The GIS has a total of 24 questions, which can be classified into five dimensions: gout concern overall, gout concern during attack, well being during attack, unmet gout treatment need, and gout medication side effects.

Intragroup analyses showed no differences regarding gout concern overall and unmet gout treatment need in all three groups (*P* > 0.05). Gout concern during the attack in the EA + DS group was reduced (*P* < 0.05). Well-being during the attack was improved in the EA + DS group (*P* < 0.05), while it was worsened in the low-dose DS group (*P* < 0.05). Gout medication side effects in both the EA + DS group and the low-dose DS group were fewer than those at baseline (*P* < 0.05). Besides, no differences were observed regarding other indicators with the intragroup analyses.

After treatment, regarding gout concern overall, there was no difference between the three groups (*P* > 0.05). Regarding gout concern and well-being during the attack, posttreatment values and variation from baseline to treatment completion in the EA + DS group had significant differences compared to those in the conventional DS group and the low-dose DS group (*P* < 0.05). Regarding unmet gout treatment need, posttreatment value and variation from baseline to treatment completion in the EA + DS group and the conventional DS group were significantly different compared to those in the low-dose DS group (*P* < 0.05). Regarding gout medication side effects, posttreatment value and variation from baseline to treatment completion in the EA + DS group had significant differences compared to those in the conventional DS group and the low-dose DS group (*P* < 0.05), except for the variation between the EA + DS group and the low-dose DS group. Besides, no differences were observed regarding other indicators with the intergroup analyses (Table 2).

### 3.4. Inflammatory Indicators

Intragroup analyses showed that the levels of CRP were lower after the treatment than those at baseline in all three groups (*P* < 0.05). After treatment, no differences were observed regarding the level of CRP and its variation from baseline to treatment completion between all three groups (*P* > 0.05).

Intragroup analyses showed that the levels of WBC and NE% in the EA + DS group and the conventional DS group were lower after treatment compared to those at baseline (*P* < 0.05). After treatment, levels of WBC, NE%, and their variation from baseline to treatment completion were greater in the EA + DS and the conventional DS group than those in the low-dose DS group (*P* < 0.05), while there were no differences between the EA + DS group and the conventional DS group (*P* > 0.05) (Table 2).

### 3.5. SUA

Intragroup analyses showed that the level of SUA was lower after the treatment compared to that at baseline in the EA + DS group (*P* < 0.05). After treatment, no differences were observed regarding the level of SUA between all three groups (*P* > 0.05), while the variation from baseline to treatment completion was greater in the EA + DS group than that in the conventional DS group and the low-dose DS group (*P* < 0.05). Besides, there were no differences between the conventional DS group and the low-dose DS group (*P* > 0.05)(Table 2).

### 3.6. Adverse Reactions

During the treatment, there were 2 cases of adverse reactions in the low-dose group, both of which had the symptom of loss of appetite. There were 4 cases of adverse reactions in the conventional DS group, including 1 case with nausea and anorexia, 1 case with anorexia, 1 case with abdominal distension, and 1 case with chest tightness. Mild symptoms were monitored and treated, and all the symptoms disappeared within 4 days. There were no adverse reactions in the EA + DS group.

### 3.7. Safety of EA

During the treatment, one patient in the EA + DS group developed local subcutaneous hematoma after acupuncture. The hematoma subsided after 2 days, and there were no other side effects or complications. All the patients in the EA + DS group had a good tolerance to the acupuncture treatment.

## 4. Discussion

Acupuncture treatment for AGA has been gradually recognized due to advantages such as anti-inflammatory and analgesic effects and the capacity to decrease the uric acid level [14]. Severe pain and activity limitation in AGA patients significantly affect their physical and mental health. However, only a few studies explored how different therapies affect the quality of life for AGA patients. Therefore, in this study, we aimed to explore whether EA combined with DS could be effective while at the same time improving the quality of life for AGA patients and reducing their dosage of analgesic drugs and adverse reactions during the treatment.

The study revealed that after a course of treatment, the clinical symptoms of joint pain, joint tenderness, joint swelling, and activity limitation in patients in the EA + DS group were improved. The performance of treatment in the EA + DS group was better than that in the low-dose DS group and was comparable to that in the conventional DS group. These results showed that combined EA and DS could synergistically relieve pain and improve the functionality of joints of AGA patients. However, the detumescence advantage of EA combined with DS was unconspicuous. It might be that the observation time was after the whole course of treatment, but a previous study found that the detumescence advantage of acupuncture was reflected immediately after a one-time treatment [18].

Through the investigation with GIS on the quality of life of AGA patients, it was found that the patients in the EA + DS group were less worried, had better health status during the attack period, and had a higher satisfaction with treatment. The “gout concern overall” is an indicator reflecting a long-term effect (usually 3 months), and thus results regarding this indicator were of little significance to the current study, which was carried out for only 1 week. In conclusion, this evaluation demonstrated the efficacy of the combined approach in treating AGA subjectively. A previous study reported a higher occurrence of depression, bipolar affective disorder, and other emotional disorders in people affected by AGA [19]. The two indicators, “gout concern during attack” and “well-being during attack,” reflected patient's psychological status, and the length of time or severity of the impact of gout on their work, mood, sleep, entertainment, social interaction, self-care ability, and activity ability [20]. Our study indicated that EA combined with DS could also improve the accompanying symptoms such as insomnia, negative emotions, and low quality of life. In addition, patients in the EA + DS group reported being less affected by the side effects of gout drugs, which was consistent with the observation that there were fewer adverse reactions for patients in the EA + DS group. DS, as a nonselective NSAID, can inhibit cyclooxygenase-1 and prostacyclin, thus causing adverse reactions in the digestive system, cardiovascular system, and kidney [21]. Thus, the current study showed that EA combined with DS could not only achieve a good curative effect but could also reduce the adverse reactions caused by the sole use of DS.

Increased counts of WBC and NE and levels of CRP are all contributing factors that facilitate urate crystals in activating downstream inflammatory factors under the action of phagocytes, thereby triggering AGA [22–24]. The anti-inflammatory effect of acupuncture on AGA may be achieved through the downregulation of interleukins and tumor necrosis factors [25, 26]. In this study, indicators including the levels of WBC, NE%, and CRP were comparable between the EA + DS group and the conventional DS group, which were better than those in the low-dose DS group. In addition, the three groups showed significant differences regarding the levels of WBC and NE% but not CRP, which might relate to the sensitivity of the indicators such as the level of CRP, which has a high sensitivity and thus, a large variation. The results regarding CRP should be comprehensively interpreted in combination with other indicators [27].

SUA is closely related to the onset and prognosis of GA. When the level of SUA in the blood exceeds its saturated solubility, the precipitated urate crystals are deposited in the joint gap, thereby triggering an inflammatory response [28]. Previous clinical studies have shown that EA can downregulate the uric acid level and its effect was superior to the DS treatment [29]. It was found that EA may achieve this effect by regulating related processes, such as purine metabolism and uric acid excretion [30, 31]. This study found that the levels of SUA were only reduced in the EA + DS group. Although the decline was not significant due to the short treatment period, it can still indicate that EA was the main factor in reducing the levels of SUA in the EA + DS combined treatment.

The efficacy of EA + DS in the treatment of AGA has been shown for the first time, but this study also has certain limitations. Firstly, owing to the characteristics of acupuncture, the acupuncturist and patients could not be blinded in this study, which might have affected the results. Secondly, these participants were recruited from only one hospital, which might lead to a lack of representativeness.

Current study used a treatment course of 5–7 days. As acupuncture treatment displays both immediate and long-term effects in AGA patients, it would be advisable to set follow-up observations to find the impact on patients' level of SUA and the recurrence rate. As the dose-effect relationship of acupuncture is also a decisive part in the curative effect of AGA treatment, the operation time or the interval between two acupuncture sessions can be further explored to optimize the therapeutic strategy during the AGA treatment [32].

## 5. Conclusion

EA combined with DS can improve AGA patients' joint pain and functional status, thus improving their quality of life. Moreover, this combined treatment can reduce levels of inflammatory markers and SUA, thus leading to fewer adverse reactions in AGA patients during treatments.

## Figures and Tables

**Figure 1:** Flow chart of the study process.

**Table 1:** Summary of demographics and baseline.

Group	EA + DS group (*n* = 30)	Low-dose group (*n* = 28)	Conventional group (*n* = 29)	*P*
Age	58.00 (46.00, 67.00)	58.00 (42.75, 62.00)	55.00 (44.00, 67.50)	0.609
BMI	25.15 ± 1.84	25.41 ± 1.55	25.86 ± 2.06	0.326
Disease duration	11.00 ± 6.68	9.86 ± 5.99	10.72 ± 6.57	0.782
VAS	7 (6, 7)	7 (6, 7)	7 (6, 7)	0.680
Joint tenderness	2 (2, 2)	2 (1.25, 3)	2 (2, 3)	0.527
Joint swelling	2 (1, 2.25)	2 (1, 2)	2 (1, 2)	0.974
Activity limitation	6.70 ± 2.15	6.43 ± 2.22	6.79 ± 2.72	0.835
GIS				
Gout concern overall	237.50 ± 75.93	255.36 ± 71.15	255.17 ± 58.77	0.525
Gout concern during attack	241.67 ± 56.98	252.68 ± 59.84	242.24 ± 41.24	0.681
Well-being during attack	634.17 ± 147.61	684.82 ± 148.66	646.55 ± 123.15	0.367
Unmet gout treatment need	157.50 ± 31.59	151.79 ± 26.29	155.17 ± 27.04	0.746
Gout medication side effects	150 (100, 156.25)	150 (100, 150)	150 (125, 162.5)	0.719
CRP	22.29 (10.49, 61.77)	24.66 (4.42, 75.50)	39.73 (12.62, 77.76)	0.543
WBC	9.22 ± 2.51	8.79 ± 3.09	9.43 ± 2.22	0.645
NE%	70.24 ± 7.86	68.86 ± 7.63	70.92 ± 9.56	0.651
SUA	490.38 ± 96.04	468.23 ± 108.44	470.78 ± 118.46	0.691

**Table 2:** Comparisons of outcome indicators and their variation from baseline to treatment completion.

Group	EA + DS group(*n* = 30)	Low-dose group (*n* = 28)	Conventionalgroup (*n* = 29)	*P*		
				EA + DS vs.low-dose	EA + DS vs.conventional	Low-dose vs.conventional
VAS	0 (0, 0)^*∗*^	1 (0, 2^*∗*^	0 (0, 0.5^*∗*^	0.001	0.692	0.005
Variation+	6 (5, 7)	5 (5, 6)	7 (6, 7)	0.026	0.512	0.004
Joint tenderness	0 (0, 0)^*∗*^	0 (0, 1^*∗*^	0 (0, 0^*∗*^	0.008	0.529	0.044
Variation+	2 (1, 2)	1 (1, 2)	2 (1, 3)	0.049	0.603	0.014
Joint swelling	0 (0, 1)^*∗*^	1 (0, 1^*∗*^	0 (0, 1^*∗*^	0.018	0.869	0.028
Variation+	2 (1, 2)	1 (0.25, 2)	2 (1, 2)	0.163		
Activity limitation	0 (0, 0)^*∗*^	0.5 (0, 2^*∗*^	0 (0, 0^*∗*^	0.001	0.916	0.001
Variation+	6.53 ± 2.21	5.21 ± 1.99	6.59 ± 2.70	0.034	0.931	0.028
GIS						
Gout concern overall	227.50 ± 73.80	260.71 ± 55.87	256.90 ± 56.65	0.092		
Variation+	0 (0, 6.25)	0 (0, 0)	0 (0, 0)	0.272		
Gout concern during attack	219.17 ± 68.76^*∗*^	262.50 ± 67.87	250.86 ± 40.91	0.008	0.048	0.470
Variation+	0 (0, 50)	0 (0, 0)	0 (0, 0)	<0.001	<0.001	0.780
Well-being during attack	570.00 ± 128.05^*∗*^	786.61 ± 146.01^*∗*^	660.34 ± 99.44	<0.001	0.007	<0.001
Variation+	25 (0, 100)	-62.5 (-231.25, 0)	−25 (−75, 62.5)	<0.001	<0.001	0.075
Unmet gout treatment need	168.33 ± 19.62	135.71 ± 31.50	157.76 ± 20.16	<0.001	0.098	0.001
Variation+	0 (-25, 0)	25 (0, 50)	0 (-12.5, 12.5)	0.003	0.374	0.042
Gout medication side effects	100 (100, 125^*∗*^	125 (125, 125^*∗*^	125 (125, 150)	0.013	<0.001	0.104
Variation+	25 (0, 50)	25 (0, 25)	0 (−12.5, 25)	0.194	0.007	0.171
CRP	4.27 (2.07, 11.51)^*∗*^	3.30 (0.83, 11.54)^*∗*^	3.86 (2.34, 9.50)^*∗*^	0.350		
Variation+	11.83 (5.45, 44.73)	12.48 (2.51, 65.00)	33.66 (2.72, 60.81)	0.527		
WBC	6.93 ± 2.25^*∗*^	8.51 ± 2.55	7.20 ± 1.76^*∗*^	0.008	0.635	0.028
Variation+	2.29 ± 2.54	0.27 ± 2.91	2.22 ± 2.39	0.004	0.917	0.006
NE%	62.43 ± 9.28^*∗*^	68.47 ± 8.72	63.26 ± 9.48^*∗*^	0.014	0.728	0.035
Variation+	7.81 ± 8.52	0.42 ± 8.34	7.66 ± 9.31	0.002	0.947	0.002
SUA	411.18 ± 83.66^*∗*^	458.76 ± 112.46	465.84 ± 89.74	0.078		
Variation+	79.19 ± 131.11	9.46 ± 111.38	4.97 ± 135.12	0.039	0.027	0.893

^+^The variation value from baseline to treatment completion. ^*∗*^There was significant difference (*P* < 0.05) in intragroup comparison from baseline to treatment completion.

## Data Availability

The data used to support the findings of this study are included within the article and available from the corresponding author upon reasonable request.

## References

[1] FitzGerald J. D., Dalbeth N., Mikuls T. (2020). 2020 American college of rheumatology guideline for the management of gout. *Arthritis Care & Research*.

[2] Roddy E., Doherty M. (2010). Epidemiology of gout. *Arthritis Research and Therapy*.

[3] Chen-Xu M., Yokose C., Rai S. K., Pillinger M. H., Choi H. K. (2019). Contemporary prevalence of gout and hyperuricemia in the United States and decadal trends: the national health and nutrition examination survey, 2007-2016. *Arthritis & Rheumatology*.

[4] Kuo C. F., Grainge M. J., Mallen C., Zhang W., Doherty M. (2015). Rising burden of gout in the UK but continuing suboptimal management: a nationwide population study. *Annals of the Rheumatic Diseases*.

[5] Annemans L., Spaepen E., Gaskin M. (2008). Gout in the UK and Germany: prevalence, comorbidities and management in general practice 2000-2005. *Annals of the Rheumatic Diseases*.

[6] Yu J.-W., Yang T.-G., Diao W.-X. (2010). Epidemiological study on hyperuricemia and gout in Foshan areas, Guangdong province. *Chinese Journal of Epidemiology*.

[7] Roddy E., Zhang W., Doherty M. (2007). Is gout associated with reduced quality of life? A case-control study. *Rheumatology*.

[8] Becker M. A., Schumacher H. R., Benjamin K. L. (2009). Quality of life and disability in patients with treatment-failure gout. *Journal of Rheumatology*.

[9] Wertheimer A., Morlock R., Becker M. A. (2013). A revised estimate of the burden of illness of gout. *Current Therapeutic Research*.

[10] Zhang S.-B., Zhang Y.-B., Liu P., Zhang W., Ma J., Wang J. (2016). Efficacy and safety of etoricoxib compared with NSAIDs in acute gout: a systematic review and a meta-analysis. *Clinical Rheumatology*.

[11] Ma K., Mi Y.-Q., Wu T. (2011). Efficacy of diclofenac sodium in pain relief after conventional radiofrequency denervation for chronic facet joint pain: a double-blind randomized controlled trial. *Pain medicine (Malden, Mass)*.

[12] Tu J.-F., Yang J.-W., Shi G. X. (2021). Efficacy of intensive acupuncture versus sham acupuncture in knee osteoarthritis: a randomized controlled trial. *Arthritis & Rheumatology*.

[13] Lv Z.-T., Shen L.-L., Zhu B. (2019). Effects of intensity of electroacupuncture on chronic pain in patients with knee osteoarthritis: a randomized controlled trial. *Arthritis Research and Therapy*.

[14] Lee W. B., Woo S. H., Min B. I., Cho S. H. (2013). Acupuncture for gouty arthritis: a concise report of a systematic and meta-analysis approach. *Rheumatology*.

[15] National Administration of Traditional Chinese Medicine (2012). *Criteria of Diagnosis and Therapeutic Effect of Diseases and Syndromes in Traditional Chinese Medicine*.

[16] Desu M. M., Raghavarao D. (1990). *Sample Size Methodology*.

[17] Hirsch J. D., Lee S. J., Terkeltaub R. (2008). Evaluation of an instrument assessing influence of gout on health-related quality of life. *Journal of Rheumatology*.

[18] Huang K. Y., Liang S., Wang J. J., Wu Y. (2015). Influence of electric-acupuncture combined with ermiao san for acute gouty arthritis model rats’ gait and joint. *Journal of liaoning University of traditional Chinese medicine*.

[19] Changchien T. C., Yen Y. C., Lin C. L., Lin M. C., Liang J. A., Kao C. H. (2015). High risk of depressive disorders in patients with gout: a nationwide population-based cohort study. *Medicine*.

[20] Pao C. H., Ko Y. (2020). An assessment of the psychometric properties of the Chinese version of the Gout Impact Scale. *Current Medical Research and Opinion*.

[21] Wilson L., Saseen J. J. (2016). Gouty arthritis: a review of acute management and prevention. *Pharmacotherapy: The Journal of Human Pharmacology and Drug Therapy*.

[22] Schiltz C., Lioté F., Prudhommeaux F. (2002). Monosodium urate monohydrate crystal-induced inflammation in vivo: quantitative histomorphometric analysis of cellular events. *Arthritis & Rheumatism*.

[23] Wessig A. K., Hoffmeister L., Klingberg A. (2022). Natural antibodies and CRP drive anaphylatoxin production by urate crystals. *Scientific Reports*.

[24] Schauer C., Janko C., Munoz L. E. (2014). Aggregated neutrophil extracellular traps limit inflammation by degrading cytokines and chemokines. *Nature Medicine*.

[25] Jin Z., Zhang Z.-Y., Jiang S.-S. (2012). Effect of acupuncture combined with medication on the contents of interleukin-1*β* and interleukin-8 in synovium of rat models of acute gouty arthritis. *Shanghai Journal of Acupuncture and moxibustion*.

[26] Long T.-L., Huang T.-J., Gao Q.-L. (2016). Effect of dredging channels and eliminating turbid acupuncture on the level of TNF-*α* in mice with acute gouty arthritis: an experimental study. *World Chinese Medicine*.

[27] Harrison M. (2015). Erythrocyte sedimentation rate and C-reactive protein. *Australian Prescriber*.

[28] Shi Y., Mucsi A. D., Ng G. (2010). Monosodium urate crystals in inflammation and immunity. *Immunological Reviews*.

[29] Zhang J.-H., Chen Y.-R., Lan K., Liyu H. U., Haibo Y. U. (2021). Clinical, anti-hyperuricemic, and pain-relief effects of five acupuncture and moxibustion therapies in acute gouty arthritis:a network meta-analysis. *Chinese General Practice*.

[30] Li R.-L., Lu X.-L., Xiong Y. (2018). Effects of combined acupuncture-drug on uric acid and xanthine oxidase activity in hyperuricemia rats with renal damage. *Shanghai Journal of Traditional Chinese Medicine*.

[31] Liu X.-F., Chen H.-Y., Wang J., Yun S. (2019). Effect of acupuncture stimulation of “Shenshu” (BL23)-Taixi (KI3) on levels of serum uric acid and renal URAT1 and OAT1 protein expression in hyperuricemia rats. *Acupuncture Research*.

[32] Shi X.-M. (2021). Study of the relationship between acupuncture dose and effect. *Acupuncture and Herbal Medicine*.

